# Biosynthesis and characterization of iron oxide nanoparticles from *Mentha spicata* and screening its combating potential against *Phytophthora infestans*

This article has been retracted.

**DOI:** 10.3389/fpls.2022.1001499

**Published:** 2022-09-26

**Authors:** Sidra Khan, Gulfam Bibi, Shazia Dilbar, Aneela Iqbal, Maaz Ahmad, Ahmad Ali, Zahid Ullah, Mariusz Jaremko, Javed Iqbal, Mohammad Ali, Ihtishamul Haq, Iftikhar Ali

**Affiliations:** ^1^Centre for Plant Sciences and Biodiversity, University of Swat, Charbagh, Khyber Pakhtunkhwa, Pakistan; ^2^Smart-Health Initiative (SHI) and Red Sea Research Center (RSRC), Division of Biological and Environmental Sciences and Engineering (BESE), King Abdullah University of Science and Technology, Thuwal, Saudi Arabia; ^3^Department of Botany, Bacha Khan University, Charsadda, Khyber Pakhtunkhwa, Pakistan; ^4^Centre for Biotechnology and Microbiology, University of Swat, Charbagh, Khyber Pakhtunkhwa, Pakistan; ^5^State Key Laboratory of Molecular Developmental Biology, Institute of Genetics and Developmental Biology, Chinese Academy of Sciences, Beijing, China

**Keywords:** *Mentha spicata*, iron chloride, iron oxide nanoparticle, calcined, *Phytophthora infestans*

## Abstract

Plant pathogens cause serious diseases to agricultural crops which lead to food insecurity in the world. To combat plant pathogens, various strategies have been developed including the use of agrochemicals. The overuse of these chemicals is now leading to the pesticide-resistant capability of pathogens. To overcome this problem, modern nanobiotechnology offers the production of alternative nano drugs. In this study, we used *Mentha spicata* for the synthesis of iron oxide nanoparticles using the green synthesis method. The synthesis of Fe_2_O_3_ NPs was confirmed through various characterizations. UV–Vis analysis detected a characteristic absorbance at the spectral range of 272 nm. The SEM micrographic analysis at various magnifications displayed circular or rod-shaped nanoparticles with a size ranging from 21 to 82 nm. The elemental EDX characterization showed intense peaks with a weight percent of 57, 34.93, and 8.07 for Fe, O, and, Cl respectively. TGA analysis showed that weight loss at 44–182, 500, and 660°C with no further modification indicates the thermal stability of iron oxide nanoparticles. FTIR spectrum of uncalined detects various bands at 3331, 1625, and 1,437 cm^−1^ for the hydroxyl group. After calcination two bands at 527 and 434 cm^−1^ were observed for Fe-O. The antimicrobial *in vitro* study showed maximum growth inhibition of *Phytophthora infestans* by the concentration of 100 μg ml^−1^ of Fe_2_O_3_-PE and Fe_2_O_3_ NPs. Therefore, this study resulted that bio-stable iron oxide nanoparticles can be used as alternative antimicrobial agents.

## Introduction

Nanotechnology is supposed to be at the forefront of the growth of nanomaterials, which are mostly used in various fields of science and technology (Abad et al., 2019; Ali et al., 2022). Nanotechnology deals with the production of nanoparticles that are useful in biological areas, particularly in drug delivery (Zahin et al., 2020). Iron is one of the most topical infrastructures because of its wide use for geological and biological processes (Abdollahi et al., 2019). Iron oxide nanoparticles are one of the prominently used particles due to their lesser toxicity and important role in ordinary use (Abbaszadeh and Hejazi, 2019). There are two types of iron oxides in nature, which are hematite and magnetite which play an exclusive role in scientific studies (Markeb et al., 2019). Iron oxide nanoparticles having a size and width of 10-100 nm played a very key role in nanotechnology (Nair et al., 2021).

The iron oxide NPs can be prepared with different methods, such as physical, chemical, and biological methods (Allafchian et al., 2019). The physical method for the synthesis of nanoparticles provides a precursor that supports the particle size in the nanometer range (Alphandéry, 2019). The chemical preparation method is very simple, and regulates the morphology, scale, and some additional properties of nanoparticles (Amanzadeh et al., 2019). In comparison to other methods, the biological process of nanoparticle synthesis is cost-effective and efficient for large-scale production (Antosova et al., 2019). Comparatively, plants provide a modest, eco-friendly, and quicker way for the synthesis of nanoparticles (Abou El-Nour et al., 2010). Plant-based synthesized nanoparticles are more effective for biological applications (Ahmad et al., 2022).

The genus *Mentha* (mints) consists of about 18 to 30 species of perennial aromatic rhizomatous herbs in the family Lamiaceae (Heylen et al., 2021). Several *Mentha* species, predominantly *M. spicata, M. pieperita, M. citrata, M. canadensis, M. longifolia* and *M. arvensis* are used in various food preparations, as kitchen spices, flavoring agents, and nutraceuticals, and are cultivated for commercial purposes for the extraction of essential oils or menthol. Menthol is among the world’s most widely utilized essential oils, worth more than 400 million US dollars (Brahmi et al., 2017). *Mentha spicata* L., commonly known as spearmint, is the most widely grown medicinal, aromatic, and flavoring herb, primarily native to Eurasia, and now cultivated in almost all parts of the world. The plant is an aromatic perennial, stoloniferous herb, reaching up to 100 cm tall, having sessile, opposite leaves, with verticellasters arranged in terminal spikes. In northern parts of Pakistan, the leaves and young shoots of *M. spicata* are used in making tea, chuttni (traditional yogurt dessert), and flavoring for a variety of dishes like corn ears, beans, etc. (Rahman et al., 2022). Leaf powder of *M. spicata* is used for the treatment of a variety of diseases including abdominal pain, stomach problems, cold, flue, fever, vomiting, bad taste, carminative, antispasmodic, diuretic, and sedative agents (Salehi et al., 2018; Mahendran et al., 2021; Rahman et al., 2022). The essential oil obtained from spearmint is used as a flavoring agent in various commercial products like cosmetics, chewing gums, toothpaste, candies, and antiemetic pills (Mahboubi, 2021). More than one hundred active phytochemicals, including phenolic acids (caffeic acid, rosemarinic acid, chlorogenic acid), flavonoids (six groups), essential oils (menthol, limonene) and lignan have been isolated from *M. spicata* leaves (15–16). Moreover, several studies have been carried out on the antimicrobial potential of *M. spicata* against a variety of bacterial and fungal pathogens. The antioxidant, anticancerous, hepatoprotective, antidiabetic, and anti-inflammatory potential of *M. spicata* is well established (Mahendran et al., 2021).

*Phytophthora infestans* is one of the important phytopathogen causing diseases to the solanaceae species, mainly potato (*Solanum tuberosum*) and tomato (*Solanum lycopersicum*; Nowicki et al., 2012). *P. infestans* belongs to the pathogenic class of oomycetes that effecting the growth of important vegetable crops (Kim and Judelson, 2003; Ali et al., 2015; Ali and Mahmood, 2015). *P. infestans* is one of the most aggressive pathogens due to its high adaptability to the host plant (Ivanov et al., 2021). *P. infestans* cause late blight disease of potato and tomato that results in postharvest yield loss worldwide (Haverkort et al., 2009). To combat *P. infestans*, humans have attempted a wide collection of strategies for more than 150 years (Ivanov et al., 2021). Including other strategies, the use of fungicides is one of the common method to lessen the growth of *P. infestans* (Pacilly et al., 2016). However, the control of this pathogen is still of immense interest because of its resistance to existing control strategies (Axel et al., 2012; Mhatre et al., 2021). Therefore, modern researchers are working on the development of new drugs to reduce the adverse effect of this pathogen (Zeyruk et al., 2022).

Keeping in view the highly medicinal applications of M. the study was designed to biosynthesize stable iron oxide nanoparticles to control the growth of *P. infestans.*

## Materials and methods

### Preparation of leaves extract and iron oxide solutions

For the preparation of leaf extract, 30 grams of *M. spicata* dried leaf powder was mixed with 100 ml deionized water in *Erlenmeyer flask* and placed on a hotplate (200 rpm stirrer) at 70 to 90°C for 30 min. The solution after cooling was filtered through Whatman Grade 1 filter paper (pore size 11 μm). For eliminating large particles of plant, the solution was centrifuged for 40 min at 4000 rpm. The obtained fine solution was stored at 4°C for further use. Next, 0.4 M iron chloride solution was prepared by dissolving 6.48 g of FeCl_3_ in 100 ml deionized water.

### Synthesis of iron oxide nanoparticles

For the synthesis of iron oxide nanoparticles, the method of Alam et al. (2019) with minor modification were employed. Concisely, 100 ml solution of FeCl_3_ (0.4 M) was mixed with equal volume (100 ml) plant extract solution. The obtained mixture was placed on a hotplate (100°C) for 30 min and observed for color change. The obtained reaction mixture after cooling was washed multiple times by pelleting and washing for 40 min in a 4,000 rpm centrifuge. Finally, the pure washed Fe_2_O_3_ NPs were obtained and dissolved in ethanol and then subjected to various characterizations.

### Characterization of Fe-oxide nanoparticles

Shimadzu pharmaspec-1700 instrument was used for UV–Vis spectrophotometric analysis. The wavelength of 200–800 nm range was set up for the detection of iron oxide nanoparticles. The band gap in the synthesized nanoparticles was defined by the formulae of (aphγ)2 = C(hγ-Eg). Where C is constant, alpha is the coefficient of absorption, and Eg is the band gap.

KYKY-EM3200 scanning electron microscope accelerating voltage of 20 kV was used to study the surface morphology of the synthesized Fe_2_O_3_ NPs. Energy dispersive X-ray (EDX) were also determined using the same instrument to describe the elemental composition of the synthesized nanoparticles.

TGA Q500 instrument was used for thermogravimetric analysis to determine the thermal stability of the synthesized Fe_2_O_3_ NPs. An alumina crucible was used for sample holding, and weight changes occurring at a constant temperature were monitored.

Bruker Optic GmbH FTIR equipped with ATR instrument was used for the identification of major chemical groups present with Fe_2_O_3_ NPs. The transmittance was recorded at the spectral range of 400–4,000 cm^−1^.

### Antimicrobial bioassay

Following Ali et al. (2015) with certain modifications, the antifungal activity against *P. infestens* were performed. The antimicrobial activity was performed over a 96 well microplate against *P. infestans* (causal agent of potato blight). Briefly, various concentrations (10, 20, 40, 60, 80, 100 μg ml^−1^) of Fe_2_O_3_ NPs were used alone and in combination with plant extract (Fe_2_O_3_-PE). The in vitro experiment was designed in triplicate and the growth inhibition was recorded in percentage. The fresh culture of *P. infestans* was obtained from the Department of Plant Pathology, University of Peshawar, Pakistan, and was grown overnight in nutrient broth. Each well of microtiter plate was adjusted with 10% V8 juice, 3,000 Zoospores, and treated with different concentrations of Fe_2_O_3_ and Fe_2_O_3_−PE NPs. The control well contains microbial suspension with distilled water. The optical density (OD) was recorded at 0 h and post 24 h and the percent growth inhibition was calculated.

## Results

### Synthesis and characterization of iron oxide nanoparticles

The reaction mixture of plant extract and iron chloride plant placed on a hotplate (100°C) and started to turn a brown color after 10 min. The solution was completely changed to a dark brown color after 30 min, which was the general indication of Fe_2_O_3_ NPs synthesis. This is due to the bio-reduction of FeCl_3_ to Fe_2_O_3_ NPs. Next, the biosynthesis of the Fe_2_O_3_ NPs was confirmed through UV–Visible spectroscopy. A maximum absorption in the UV/visible spectrum occurred at 272 nm, suggesting the synthesis of Fe_2_O_3_ NPs (Figure 1). The band gap energy calculated for the synthesized nanoparticles was found to be 2.23 eV.

**Figure 1:** UV–V is analysis of the synthesized iron oxide nanopracticles.

### Scanning electron microscopy

The scanning electron microscopic observation of the synthesized Fe_2_O_3_ NPs using various magnifications power gives the morphology, sticking, and dispersion details. The size of the synthesized nanoparticles was ranging from 21 to 82 nm. The surface morphology of nanoparticles showed irregularly shaped particles due to the changed reactant concentration of iron chloride and plant extract. However, most of the synthesized Fe_2_O_3_ NPs were found to be circular and rod shaped. The SEM analysis showed strong dispersion that enhanced the nanoparticles characteristics (Figure 2).

**Figure 2:** SEM micrographs of iron oxide nanopracticles.

### Energy dispersive X-ray

The EDX elemental diffraction analysis confirmed the sample composition through a high-intensity peak. The first EDX intensity peak indicated the presence of iron and the second intensity peak showed the existence of oxygen that further confirms the preparation of iron oxide nanoparticles. Further, a wide intensity peak of chlorine was found that was due to the chloride present in the iron chloride solution. Iron is around 57 percent by weight, oxygen is 34.93 percent and chlorine is 8.07 percent, according to the EDX peak analysis. Moreover, no other peaks were observed that confirmed the synthesis of pure iron oxide nanoparticles (Figure 3).

**Figure 3:** EDX elemental characterization of the biosynthesized iron oxide nanopracticles.

### Thermogravimetric analysis of Fe_2_O_3_NPs

The thermogravimetric analysis was carried out from room temperature to 800°C. The weight loss happens at distinct times as the temperature increases. The first weight loss happens between 44 and 182°C which was about 5.56 percent due to the elimination of water from the surface of Fe_2_O_3_ NPs. As the temperature reaches up to 500°C, another weight loss of 3.04 percent was detected due to the removal of organic compounds found in the nanoparticles. Similarly, a minor weight loss of 1.38 percent was observed at 660°C due to the transformation step of the Fe_2_O_3_ NPs. Next, no further modifications were observed after 660°C, suggesting that the synthesized Fe_2_O_3_ NPs were extremely thermally stable (Figure 4).

**Figure 4:** TGA of biosynthesized iron oxide nanopracticles.

### Fourier transform infrared spectroscopy

FTIR spectrum showed the uncalcined and calcined peaks at various positions. Uncalcined nanoparticles identify two bands located at 3331 cm^−1^ and 1,625 cm^−1^ for the stretching and blending vibration of water molecules or hydroxyl group. This indicates the presence of a small amount of water molecules or certain hydroxide groups on the surface of nanoparticles. This was found because the product was synthesized in an aqueous solution. A band at 1437 cm^−1^ was observed which was assigned for the CH3 deformation. The FTIR spectrum of nanoparticles at 700°C synthesized by the precipitation method detects no band associated with the hydroxyl group (OH). After calcination, the complete organic species have been extracted for the particles. The calcined spectrum showed bands located at 527 cm^−1^ and 434 cm^−1^, which can be attributed to the vibration of Fe_2_O_3_ NPs (Figure 5).

**Figure 5:** FTIR analysis of the iron oxide nanopracticles.

### Antimicrobial bioassay

The concentration of 100 μg ml^−1^ of Fe_2_O_3_ NPs alone and in combination with plant extract (Fe_2_O_3_-PE) showed maximum inhibition of the growth of *P. infestans*. The Fe_2_O_3_ and Fe_2_O_3_-PE NPs at 100 μg ml^−1^ inhibited the growth by 90 and 98 percent, respectively. Our result showed that Fe_2_O_3_ NPs in combination with plant extract is significant against *P. infestans*. The control concentration treatment showed no inhibition of the growth of *P. infestans* (Figure 6).

**Figure 6:** Antimicrobial bioassay showing the inhibitory growth effects of *P. inseftence* in response to difference concentration of Fe_2_O_3_ NPs alone and in combination with plant extract (Fe_2_O_3_-PE).

## Discussion

Due to its non-hazardous nature, iron oxide nanoparticles have been used by researchers for various medical and industrial applications (Ling and Hyeon, 2013). The biological synthesis of Fe_2_O_3_ NPs is of immense interest because it is cost-effective and non-toxic to humans (Kharey et al., 2022). Iron oxide nanoparticles perform numerous applications against biotic and abiotic stresses and play an important role in various medical and biological fields (Irum et al., 2020). The antimicrobial applications of iron oxide nanoparticles provide a significant solution to control plant pathogens (Parveen et al., 2018). Previous studies report the effective synthesis of bio-stable Fe_2_O_3_ NPs which were used for various biological applications (Lam et al., 2013; Rajiv et al., 2017). Medicinal plants are considered to be the core agents for the synthesis of iron oxide nanoparticles (Hernández-Hernández et al., 2020; Jamzad and Kamari, 2020). Plants contain various secondary compounds such as phenols, flavonoids, glycosides, alkaloids, etc., which act as a reducing and capping agent for the synthesis of stable metal oxide nanoparticles (Ishak et al., 2019; Gebre, 2022). Plant secondary constituents provide stability to nanoparticles and offer a feasible way for large-scale nanoparticle synthesis (Saif et al., 2016; Küünal et al., 2018). Recent studies report the efficient synthesis of stable iron oxide nanoparticles using plant extracts (Demirezen et al., 2019; Abdullah et al., 2020; Lakshminarayanan et al., 2021).

In the present study, we showed the plant extract of *M. spicata* has effectively synthesized stable Fe_2_O_3_ NPs. The reduction of iron chloride in the presence of aqueous plant extract was generally observed by the color change of the reaction mixture. The UV–Vis surface plasmon resonance peak at the wavelength of 272 nm was detected that revealed nanoparticle synthesis. Similarly, no other UV–Vis absorption peak was detected that indicated the formation of pure nanoparticles. The surface morphology of the produced nanoparticles was observed during SEM micrographs. The observed particles were of irregular shape but most of them were rod or circular having strong dispersion with a size in the range of 21 to 82 nm. The EDX study indicated the high-intensity peaks of iron, oxygen, and chloride. The EDX analysis showed a clear elemental composition where no undesirable element was detected thus confirming the complete pure Fe_2_O_3_ nanoparticles synthesis. The FTIR analysis for both uncalcined and calcined iron oxide nanoparticles was effectively observed. The obtained results showed various bands however the presence of two bands was noticed at 527 and 434 cm^−1^ after calcination. These showed that the calcined nanoparticles have no biological constituent hence they are purer than uncalcined particles. The antimicrobial bioassay showed strong inhibition of the growth of *P. infestans* by 100 μg ml^−1^. The highest inhibition percent recorded by the Fe_2_O_3_-PE nanoparticles was due to the presence of plant extract.

The synthesis of Fe_2_O_3_ NPs during UV–Visible analysis showed a similar pattern to those previously reported (Madubuonu et al., 2020). The SEM and EDX results were compared with previous studies which showed matching observations of Fe_2_O_3_ NPs (Alam et al., 2019; Sudhakar et al., 2022). The FTIR characterization was complete corresponding to previously reported data (Ali et al., 2021). Moreover, the obtained antimicrobial results were correlated with the previous literature and were completely corresponding (Seddighi et al., 2017; Devi et al., 2019). Our results regarding synthesis, characterization, and antimicrobial activity showed the formation of efficient and stable Fe_2_O_3_ NPs showing significant antimicrobial potential.

## Conclusion

In this study, we showed the biosynthesis of iron oxide nanoparticles using the extract of *M. spicata*. The synthesized nanoparticles were studied through different characterization techniques. Our findings revealed the significant biosynthesis of iron oxide nanoparticles from *M. spicata*. The study showed that the prepared nanoparticles were highly stable because of the capping layers provided by plant extract. Moreover, the prepared Fe_2_O_3_ NPs strongly inhibited the growth of *P. infestans*. These findings determine that Fe_2_O_3_ NPs have the potential to control the growth of *P. infestans*. Therefore, this study has set an optimized baseline for the biosynthesis of stable antifungal Fe_2_O_3_ NPs using plant extracts. However, due to the complex mechanism of antimicrobial activity further studies should examine the effects of Fe_2_O_3_ NPs against plant pathogens.

## Data availability statement

The original contributions presented in the study are included in the article/supplementary material, further inquiries can be directed to the corresponding authors.

## Author contributions

SD, MoA, and AA conceived and designed the research. SK, GB, and IH conducted the research. Interpretation of the results was done by ZU, MJ, and MaA. IA, JI, and MJ wrote the final draft of manuscript. AI, AA, ZU, and MaA checked the final content of the manuscript. All authors read and accepted the final version of the manuscript.

## Conflict of interest

The authors declare that the research was conducted in the absence of any commercial or financial relationships that could be construed as a potential conflict of interest.

## Publisher’s note

All claims expressed in this article are solely those of the authors and do not necessarily represent those of their affiliated organizations, or those of the publisher, the editors and the reviewers. Any product that may be evaluated in this article, or claim that may be made by its manufacturer, is not guaranteed or endorsed by the publisher.

## References

[ref1] AbadT. S.ZoidlG.Ghafar-ZadehE. (2019). A multidisciplinary approach toward high throughput label-free cytotoxicity monitoring of superparamagnetic iron oxide nanoparticles. Bioengineering 6:52. doi: 10.3390/bioengineering6020052, PMID: 31185664PMC6631604

[ref2] AbbaszadehM.HejaziP. (2019). Metal affinity immobilization of cellulase on Fe3O4 nanoparticles with copper as ligand for biocatalytic applications. Food Chem. 290, 47–55. doi: 10.1016/j.foodchem.2019.03.117, PMID: 31000055

[ref3] AbdollahiZ.Taheri-KafraniA.BahraniS. A.KajaniA. A. (2019). PEGAylated graphene oxide/superparamagnetic nanocomposite as a high-efficiency loading nanocarrier for controlled delivery of methotrexate. J. Biotechnol. 298, 88–97. doi: 10.1016/j.jbiotec.2019.04.006, PMID: 30986517

[ref4] AbdullahJ. A. A.EddineL. S.AbderrhmaneB.Alonso-GonzálezM.GuerreroA.RomeroA. (2020). Green synthesis and characterization of iron oxide nanoparticles by *Pheonix dactylifera* leaf extract and evaluation of their antioxidant activity. Sustain. Chem. Pharm. 17:100280. doi: 10.1016/j.scp.2020.100280

[ref5] Abou El-NourK. M.EftaihaA. A.Al-WarthanA.AmmarR. A. (2010). Synthesis and applications of silver nanoparticles. Arab. J. Chem. 3, 135–140. doi: 10.1016/j.arabjc.2010.04.008

[ref300] AhmadM.AliA.UllahZ.SherH.DaiD-Q.AliM.. (2022). Biosynthesized silver nanoparticles using Polygonatum geminiflorum efficiently control fusarium wilt disease of tomato. Front. Bioeng. Biotechnol. 10:988607. doi: 10.3389/fbioe.2022.98860736159677PMC9493356

[ref6] AlamT.KhanR. A. A.AliA.SherH.UllahZ.AliM. (2019). Biogenic synthesis of iron oxide nanoparticles via *Skimmia laureola* and their antibacterial efficacy against bacterial wilt pathogen *Ralstonia solanacearum*. Mater. Sci. Eng. C 98, 101–108. doi: 10.1016/j.msec.2018.12.117, PMID: 30812984

[ref7] AliA. A.AhmedI. S.ElfikyE. M. (2021). Auto-combustion synthesis and characterization of iron oxide nanoparticles (α-Fe2O3) for removal of lead ions from aqueous solution. J. Inorg. Organomet. Polym. Mater. 31, 384–396. doi: 10.1007/s10904-020-01695-3

[ref8] AliI.KhanA.AliA.UllahZ.DaiD.KhanN.. (2022). Iron and zinc micronutrients and soil inoculation of *Trichoderma harzianum* enhance wheat grain quality and yield. Front. Plant Sci. 13:960948. doi: 10.3389/fpls.2022.96094836160992PMC9490233

[ref9] AliM.KimB.BelfieldK. D.NormanD.BrennanM.AliG. S. (2015). Inhibition of *Phytophthora parasitica* and *P. capsici* by silver nanoparticles synthesized using aqueous extract of *Artemisia absinthium*. Phytopathology 105, 1183–1190. doi: 10.1094/PHYTO-01-15-0006-R, PMID: 25871856

[ref10] AliI.MahmoodT. (2015). Identification and analysis of regulatory elements in the germin and germin-like proteins family promoters in rice. Turk. J. Bot. 39, 389–400. doi: 10.3906/bot-1405-48

[ref11] AliI.SardarZ.RasheedA.MahmoodT. (2015). Molecular characterization of the puroindoline-a and b alleles in synthetic hexaploid wheats and in silico functional and structural insights into Pina-D1. J. Theor. Biol. 376, 1–7. doi: 10.1016/j.jtbi.2015.04.001, PMID: 25865523

[ref12] AllafchianA.MousaviZ. S.HosseiniS. S. (2019). Application of cress seed musilage magnetic nanocomposites for removal of methylene blue dye from water. Int. J. Biol. Macromol. 136, 199–208. doi: 10.1016/j.ijbiomac.2019.06.083, PMID: 31201917

[ref13] AlphandéryE. (2019). Biodistribution and targeting properties of iron oxide nanoparticles for treatments of cancer and iron anemia disease. Nanotoxicology 13, 573–596. doi: 10.1080/17435390.2019.1572809, PMID: 30938215

[ref14] AmanzadehE.EsmaeiliA.AbadiR. E. N.KazemipourN.PahlevanneshanZ.BeheshtiS. (2019). Quercetin conjugated with superparamagnetic iron oxide nanoparticles improves learning and memory better than free quercetin via interacting with proteins involved in LTP. Sci. Rep. 9, 1–19. doi: 10.1038/s41598-019-43345-w31053743PMC6499818

[ref15] AntosovaA.BednarikovaZ.KonerackaM.AntalI.MarekJ.KubovcikovaM.. (2019). Amino acid functionalized superparamagnetic nanoparticles inhibit lysozyme amyloid fibrillization. Chem. Eur. J. 25, 7501–7514. doi: 10.1002/chem.201806262, PMID: 30958585

[ref16] AxelC.ZanniniE.CoffeyA.GuoJ.WatersD. M.ArendtE. K. (2012). Ecofriendly control of potato late blight causative agent and the potential role of lactic acid bacteria: a review. Appl. Microbiol. Biotechnol. 96, 37–48. doi: 10.1007/s00253-012-4282-y, PMID: 22864968

[ref17] BrahmiF.KhodirM.MohamedC.PierreD. (2017). Chemical composition and biological activities of *Mentha* species. Aromat. Medic. Plants Back Nat. 10, 47–79. doi: 10.5772/67291

[ref18] DemirezenD. A.YıldızY. Ş.YılmazŞ.YılmazD. D. (2019). Green synthesis and characterization of iron oxide nanoparticles using *Ficus carica* (common fig) dried fruit extract. J. Biosci. Bioeng. 127, 241–245. doi: 10.1016/j.jbiosc.2018.07.024, PMID: 30348486

[ref19] DeviH. S.BodaM. A.ShahM. A.ParveenS.WaniA. H. (2019). Green synthesis of iron oxide nanoparticles using *Platanus orientalis* leaf extract for antifungal activity. Green Process Synth. 8, 38–45. doi: 10.1515/gps-2017-0145

[ref20] GebreS. H. (2022). Bio-inspired synthesis of metal and metal oxide nanoparticles: the key role of phytochemicals. J. Clust. Sci. 33, 1–40. doi: 10.1007/s10876-022-02276-9

[ref21] HaverkortA. J.StruikP. C.VisserR. G. F.JacobsenE. J. P. R. (2009). Applied biotechnology to combat late blight in potato caused by *Phytophthora infestans*. Potato Res. 52, 249–264. doi: 10.1007/s11540-009-9136-3

[ref22] Hernández-HernándezA. A.Aguirre-ÁlvarezG.Cariño-CortésR.Mendoza-HuizarL. H.Jiménez-AlvaradoR. (2020). Iron oxide nanoparticles: synthesis, functionalization, and applications in diagnosis and treatment of cancer. Chem. Pap. 74, 3809–3824. doi: 10.1007/s11696-020-01229-8

[ref23] HeylenO. C.DebortoliN.MarescauxJ.OlofssonJ. K. (2021). A revised phylogeny of the Mentha spicata clade reveals cryptic species. Plan. Theory 10:819. doi: 10.3390/plants10040819, PMID: 33924227PMC8074783

[ref24] IrumS.JabeenN.AhmadK. S.ShafiqueS.KhanT. F.GulH.. (2020). Biogenic iron oxide nanoparticles enhance callogenesis and regeneration pattern of recalcitrant *Cicer arietinum* L. PLoS One 15:e0242829. doi: 10.1371/journal.pone.0242829, PMID: 33259506PMC7707474

[ref25] IshakN. M.KamarudinS. K.TimmiatiS. N. (2019). Green synthesis of metal and metal oxide nanoparticles via plant extracts: an overview. Mater. Res. Express 6:112004. doi: 10.1088/2053-1591/ab4458

[ref26] IvanovA. A.UkladovE. O.GolubevaT. S. (2021). *Phytophthora infestans*: an overview of methods and attempts to combat late blight. J. Fungi 7:1071. doi: 10.3390/jof7121071, PMID: 34947053PMC8707485

[ref27] JamzadM.KamariB. M. (2020). Green synthesis of iron oxide nanoparticles by the aqueous extract of *Laurus nobilis* L. leaves and evaluation of the antimicrobial activity. J. Nanostructure Chem. 10, 193–201. doi: 10.1007/s40097-020-00341-1

[ref28] KhareyP.IndoliyaA.GuptaR.PoddarR.SharmaD.GuptaS. (2022). Near-infrared active superparamagnetic iron oxide nanoparticles for magnetomotive optical coherence tomography imaging and magnetic hyperthermia therapeutic applications. J. Magn. Magn. Mater. 549:169038. doi: 10.1016/j.jmmm.2022.169038

[ref29] KimK. S.JudelsonH. S. (2003). Sporangium-specific gene expression in the oomycete phytopathogen *Phytophthora infestans*. Eukaryot. Cell 2, 1376–1385. doi: 10.1128/EC.2.6.1376-1385.2003, PMID: 14665470PMC326645

[ref30] KüünalS.RauwelP.RauwelE. (2018). “Plant extract mediated synthesis of nanoparticles,” in Emerging Applications of Nanoparticles and Architecture Nanostructures eds. BarhoumA.MakhloufA. S. H. (Amsterdam: Elsevier), 411–446. doi: 10.1016/B978-0-323-51254-1.00014-2

[ref31] LakshminarayananS.ShereenM. F.NiraimathiK. L.BrindhaP.ArumugamA. (2021). One-pot green synthesis of iron oxide nanoparticles from *Bauhinia tomentosa*: characterization and application towards synthesis of 1, 3 diolein. Sci. Rep. 11, 1–13. doi: 10.1038/s41598-021-87960-y33883589PMC8060310

[ref32] LamT.PouliotP.AvtiP. K.LesageF.KakkarA. K. (2013). Superparamagnetic iron oxide based nanoprobes for imaging and theranostics. Adv. Colloid Interf. Sci. 199-200, 95–113. doi: 10.1016/j.cis.2013.06.00723891347

[ref33] LingD.HyeonT. (2013). Chemical design of biocompatible iron oxide nanoparticles for medical applications. Small 9, 1450–1466. doi: 10.1002/smll.201202111, PMID: 23233377

[ref34] MadubuonuN.AisidaS. O.AhmadI.BothaS.ZhaoT. K.MaazaM.. (2020). Bio-inspired iron oxide nanoparticles using *Psidium guajava* aqueous extract for antibacterial activity. Appl. Phys. A Mater. Sci. Process. 126, 1–8. doi: 10.1007/s00339-019-3249-6

[ref35] MahboubiM. (2021). Mentha spicata L. essential oil, phytochemistry and its effectiveness in flatulence. J. Tradit. Complement. Med. 11, 75–81. doi: 10.1016/j.jtcme.2017.08.011, PMID: 33728265PMC7936090

[ref36] MahendranG.VermaS. K.RahmanL. U. (2021). The traditional uses, phytochemistry and pharmacology of spearmint (*Mentha spicata* L.): a review. J. Ethnopharmacol. 278:114266. doi: 10.1016/j.jep.2021.114266, PMID: 34087400

[ref37] MarkebA. A.Llimós-TuretJ.FerrerI.BlánquezP.AlonsoA.SánchezA.. (2019). The use of magnetic iron oxide based nanoparticles to improve microalgae harvesting in real wastewater. Water Res. 159, 490–500. doi: 10.1016/j.watres.2019.05.023, PMID: 31128473

[ref38] MhatreP. H.LekshmananD. K.PalanisamyV. E.BairwaA.SharmaS. (2021). Management of the late blight (*Phytophthora infestans*) disease of potato in the southern hills of India. J. Phytopathol. 169, 52–61. doi: 10.1111/jph.12958

[ref39] NairG. M.SajiniT.MathewB. (2021). Advanced green approaches for metal and metal oxide nanoparticles synthesis and their environmental applications. Talanta Open 5:100080. doi: 10.1016/j.talo.2021.100080

[ref40] NowickiM.FooladM. R.NowakowskaM.KozikE. U. (2012). Potato and tomato late blight caused by *Phytophthora infestans*: an overview of pathology and resistance breeding. Plant Dis. 96, 4–17. doi: 10.1094/PDIS-05-11-0458, PMID: 30731850

[ref41] PacillyF. C.GrootJ. C.HofstedeG. J.SchaapB. F.van BuerenE. T. L. (2016). Analysing potato late blight control as a social-ecological system using fuzzy cognitive mapping. Agron. Sustain. Dev. 36, 1–18. doi: 10.1007/s13593-016-0370-1

[ref42] ParveenS.WaniA. H.ShahM. A.DeviH. S.BhatM. Y.KokaJ. A. (2018). Preparation, characterization and antifungal activity of iron oxide nanoparticles. Microb. Pathog. 115, 287–292. doi: 10.1016/j.micpath.2017.12.068, PMID: 29306005

[ref43] RahmanS. U.UllahZ.AliA.AzizM. A.AlamN.SherH.. (2022). Traditional knowledge of medicinal flora among tribal communities of Buner Pakistan. Phytomed. Plus 2:100277. doi: 10.1016/j.phyplu.2022.100277

[ref44] RajivP.BavadharaniB.KumarM. N.VanathiP. (2017). Synthesis and characterization of biogenic iron oxide nanoparticles using green chemistry approach and evaluating their biological activities. Biocatal. Agric. Biotechnol. 12, 45–49. doi: 10.1016/j.bcab.2017.08.015

[ref45] SaifS.TahirA.ChenY. (2016). Green synthesis of iron nanoparticles and their environmental applications and implications. Nano 6:209. doi: 10.3390/nano6110209, PMID: 28335338PMC5245755

[ref46] SalehiB.Stojanović-RadićZ.MatejićJ.SharopovF.AntolakH.KręgielD.. (2018). Plants of genus *Mentha*: from farm to food factory. Plan. Theory 7:70. doi: 10.3390/plants7030070, PMID: 30181483PMC6161068

[ref47] SeddighiN. S.SalariS.IzadiA. R. (2017). Evaluation of antifungal effect of iron-oxide nanoparticles against different *Candida* species. IET Nanobiotechnol. 11, 883–888. doi: 10.1049/iet-nbt.2017.0025

[ref48] SudhakarC.PoonkothaiM.SelvankumarT.SelvamK. (2022). Facile synthesis of iron oxide nanoparticles using *Cassia auriculata* flower extract and accessing their photocatalytic degradation and larvicidal effect. J. Mater. Sci. Mater. Electron. 33, 11434–11445. doi: 10.1007/s10854-022-08116-w

[ref49] ZahinN.AnwarR.TewariD.KabirM.SajidA.MathewB.. (2020). Nanoparticles and its biomedical applications in health and diseases: special focus on drug delivery. Environ. Sci. Pollut. Res. 27, 19151–19168. doi: 10.1007/s11356-019-05211-0, PMID: 31079299

[ref50] ZeyrukV. N.VasilievaS. V.BelovG. L.DerevyaginaM. K.BogoslovskayaO. A.OlkhovskayaI. P.. (2022). A boost to integrated management of certain potato diseases using metal nanoparticles. Potato Res. 65, 273–288. doi: 10.1007/s11540-021-09518-9

